# Predictive Value of the HEART Score Combined with Hypersensitive C-Reactive Protein for 30 d Adverse Cardiovascular Events in Patients with Acute Chest Pain

**DOI:** 10.1155/2022/3606169

**Published:** 2022-11-10

**Authors:** Maosheng Lin, Louwei Zhang, Xuhua Tang, Yejiang Tang

**Affiliations:** Department of Emergency Medicine, Zhuji Affiliated Hospital of Wenzhou Medical University, Zhuji, Zhejiang 311800, China

## Abstract

**Purpose:**

This study aimed to explore the predictive value of the HEART score combined with hypersensitive C-reactive protein (hs-CRP) for 30 d major adverse cardiovascular events (MACEs) in patients with acute chest pain.

**Methods:**

103 patients with acute chest pain admitted to the emergency department of our hospital from May 2020 to May 2022 were selected as the study subjects. The patients' HEART score and plasma hs-CRP level were recorded. The patients were followed up for 30 d to observe whether MACE occurred.

**Results:**

Among 103 patients with acute chest pain, MACE occurred in 8 cases within 30 d of follow-up, and the probability of MACE was 7.76%. There was a statistically significant difference in 30 d MACE risk among patients with different HEART score stratification (*P* < 0.05). The age, HEART score, and hs-CRP levels of patients in the MACE group were higher than those in the non-MACE group (*P* < 0.05). The HEART score and the hs-CRP level were independent risk factors for 30 d MACE in patients with acute chest pain (*P* < 0.05). The AUC of the HEART score combined with hs-CRP in the occurrence of 30 d MACE in patients with acute chest pain was 0.901, which was significantly higher than 0.720 and 0.758 of single detection.

**Conclusion:**

The HEART score combined with hs-CRP can better predict the occurrence of 30 d MACE in patients with acute chest pain.

## 1. Introduction

Acute chest pain is a clinical emergency, and its incidence accounts for 5%–20% of patients in emergency medicine and even 20%–30% in large tertiary hospitals [1]. Acute chest pain can be divided into cardiogenic and noncardiogenic chest pain, of which, acute cardiogenic chest pain is one of the main types [2]. Acute cardiogenic chest pain is rapid in onset and progression and has a complex etiology, variable clinical manifestations, and high risk factors, which may lead to malignant events such as heart failure and arrhythmias, and even disability or death [3, 4]. It has been reported that the incidence of major adverse cardiovascular events (MACEs) in patients with acute chest pain is higher than that in the normal population. Therefore, timely identification of the risk of chest pain and assessment of the patient's prognosis are conducive to guiding clinical treatment and improving the survival rate and are of great value for improving the prognosis [5]. In addition, due to the lack of accurate symptom manifestations of acute chest pain and the mostly atypical ECG, the optimal treatment time is easily missed, and sudden cardiac events are possible [6]. Therefore, how to rapidly predict MACE in acute chest pain has become an urgent clinical problem to be explored.

In order to quickly differentiate between chest pain categories and assess the degree of risk, emergency physicians in China and abroad have developed many acute chest pain scoring systems to make accurate treatment decisions and improve patients' quality of life as early as possible [7, 8]. The HEART score is simple, fast, convenient, and economical. It can be performed within 1 hour after patients with chest pain receive treatment, helping doctors estimate the patient's condition as early as possible [9, 10]. C-reactive protein (CRP) is used as a monitoring indicator for acute illnesses and can quickly respond to the severity of infection, inflammation, and tissue damage [11]. Hypersensitive CRP (hs-CRP) is an acute temporal protein produced by the human body in response to microbial invasion or tissue inflammation and is synthesized by the human liver [12]. hs-CRP is more than 10 times more sensitive than CRP, and assessing hs-CRP levels can help doctors estimate the risk of cardiovascular disease in patients.

At present, there are few clinical studies on the predictive value of the HEART score combined with hs-CRP on 30 d MACE in patients. Therefore, in this study, 103 patients with acute chest pain were selected to observe the occurrence of 30 d MACE and to analyze the relationship between the HEART score, hs-CRP, and MACE.

## 2. Materials and Methods

### 2.1. Research Objects

103 patients with acute chest pain admitted to the emergency department of our hospital from May 2020 to May 2022 were selected as the study subjects. Inclusion criteria were as follows: presented with chest pain as the main symptom; chest pain onset within 12 h; age ≥ 18 years; complete medical records and able to complete follow-up. Exclusion criteria were as follows: chest pain caused by trauma; systemic pain due to rheumatic diseases involving the chest; liver and kidney insufficiency; combined with malignant tumors, infectious diseases or psychiatric diseases; a recent history of heart valve disease, cardiomyopathy, myocarditis, etc.

### 2.2. Research Methods

All patients were treated symptomatically on admission according to their condition. ① After admission, a risk score was assigned to all enrolled patients based on the HEART scoring system. The total score was 10 points, with 0∼3 points being the low-risk group (*n* = 20), 4∼6 points being the moderate-risk group (*n* = 44), and 7∼10 points being the high-risk group (*n* = 39). The HEART scoring system is shown in Table 1. ② After patients were admitted to the hospital, 4 ml of peripheral venous blood was drawn, anticoagulated with sodium citrate, and centrifuged at 3000 r/min. Plasma was separated and stored at −70°C. Plasma hs-CRP levels were measured by the immunoturbidimetric assay. ③ Patients were followed up for 30 d after discharge using outpatient review, door-to-door face-to-face visits, or telephone. The occurrence of MACE within 30 d was recorded, and MACE included all-cause death, myocardial infarction, unstable angina, emergency revascularization, cardiogenic shock, and cardiac arrest/ventricular fibrillation.

### 2.3. Statistical Methods

SPSS 20.0 software was used for analysis. The measurement data were expressed as the mean ± SD, and the *t*-test was used for comparison. Count data were expressed as rates, and the *χ*^2^ test was used for comparison. Logistic regression models were used to analyze risk factors. The AUC in the subject's ROC was used to express the predictive value. The difference was considered significant at *P* < 0.05.

## 3. Results

### 3.1. Occurrence of 30 d MACE in Patients with Acute Chest Pain

Among 103 patients with acute chest pain, MACE occurred in 8 cases within 30 d of follow-up, and the probability of MACE was 7.76%. Of these, all-cause death occurred in 6 cases, myocardial infarction occurred in 1 case, and unstable angina occurred in 1 case.

### 3.2. Occurrence of 30 d MACE in Patients with Different HEART Scores

There was a statistically significant difference in 30 d MACE risk among patients with different HEART score stratification (*P* < 0.05), as shown in Table 2.

### 3.3. Comparison of Clinical Data between the Two Groups

The age, HEART score, and hs-CRP levels of patients in the MACE group were higher than those in the non-MACE group (*P* < 0.05). There was no statistically significant difference between the remaining clinical information of the two groups (*P* > 0.05), as shown in Table 3.

### 3.4. Risk Factors for 30 d MACE in Patients with Acute Chest Pain

Multifactorial logistic analysis showed that the HEART score and the hs-CRP level were independent risk factors for 30 d MACE in patients with acute chest pain (*P* < 0.05), as shown in Table 4.

### 3.5. Predictive Value of Different Indicators for 30 d MACE in Patients with Acute Chest Pain

The AUC of the HEART score in predicting 30 d MACE in patients with acute chest pain was 0.720. The AUC of hs-CRP in predicting 30 d MACE in patients with acute chest pain was 0.758. The AUC of the HEART score combined with hs-CRP in predicting 30 d MACE in patients with acute chest pain was 0.901, as shown in Table 5 and Figure 1.

## 4. Discussion

Acute chest pain is one of the more dangerous diseases in the emergency department and is a pain that occurs in the chest or radiates from other parts of the body to the chest [13]. The causes of acute chest pain are many and involve multiple organs and systems, commonly including chest boils and carbuncles, herpes zoster, trauma, pneumothorax, myocarditis, and abdominal diseases [14]. For patients with acute cardiogenic chest pain, taking active treatment and predicting the occurrence of MACE can obviously improve the prognosis of patients and then improve the survival rate of patients [15]. Therefore, there is great clinical value in using a simple, practical, quick, and accurate method to assess the prognosis of patients with acute chest pain.

The HEART score is a nonspecific scoring system that does not require inclusion or exclusion criteria for patients with chest pain, and the items of the score are easy to collect data and less difficult to calculate, which facilitates daily use by clinical workers [16]. Unlike other chest pain scoring systems, the HEART score includes patient history, ECG, age, risk factors, and troponin levels, emphasizing the combination of ECG and troponin levels, which is more accurate than conventional assessment methods [17]. At the same time, the HEART score assesses different independent risk components in patients with acute chest pain without the need for clear evidence of acute coronary syndromes and can identify patients' condition and prognosis as soon as possible [18]. The HEART score can be evaluated within 1 hour after the patient is admitted to the hospital, so the HEART score is suitable for patients diagnosed with urgent intervention and meets the requirement of clinical emergency treatment [19]. The HEART score can quickly and effectively communicate the risks associated with acute chest pain, allowing for a quick understanding of the patient's risk level and helping physicians intervene according to the patient's risk level [20]. In this study, the incidence of 30 d MACE in the HEART high-risk group was higher than that in the moderate-risk group and the low-risk group, and the HEART score was an independent risk factor for 30 d MACE in patients with acute chest pain. The results suggest that the HEART score has good efficacy for assessing the occurrence of MACE in patients with chest pain in the short term.

It has been reported that the occurrence of acute cardiogenic chest pain is closely related to the body's inflammatory response and coagulation formation [21]. As an inflammatory factor, CRP inhibits neovascularization by promoting endothelial cell apoptosis. Since CRP reflects macrophage activity and plaque rupture correlates with macrophage activity, CRP is associated with atherosclerotic plaque vulnerability [22]. CRP activates the complement system and produces complement terminal complexes that cause direct damage to the intima, which in turn leads to vasospasm and unstable plaque rupture. Boncler M et al. showed that plasma concentrations of CRP are relatively low in a healthy population, while plasma CRP levels are significantly increased when the organism is under inflammation, stress, or trauma [23]. At the same time, changes in CRP levels are closely associated with cardiovascular disease risk factors such as diabetes, hypertension, and hyperlipidemia. In clinical, compared to CRP, hs-CRP can reflect cardiovascular inflammation more sensitively and accurately and is not affected by taking food and circadian rhythms [24]. Under normal circumstances, the concentration of hs-CRP in plasma was in a stable state for a long period. After tissue damage in patients, hs-CRP concentration could rise rapidly and be detected in blood within 6–8 h and reached the peak at 24–48 h. [25]. Caselli C et al. concluded that hs-CRP, as a marker of inflammation, is able to monitor the severity of disease and has high predictive accuracy for the development of coronary artery disease in patients with chronic chest pain [26]. We found that hs-CRP levels in the MACE group were higher, and the level of hs-CRP can predict the occurrence of MACE in patients with acute chest pain for 30 d.

Only troponin is included in the HEART scoring system, which shows poor specificity. Therefore, the addition of another biomarker above the cardiac score has a positive effect on improving the evaluation of acute chest pain. In addition, hs-CRP has good specificity but relatively poor sensitivity, and the predictive value of a single test is not high, so it has good significance to combine the two. In view of the limitations of the HEART score and hs-CRP alone in predicting the short-term prognosis, we applied the combination of the HEART score and hs-CRP in prognostic assessment. The AUC of the HEART score combined with hs-CRP in the occurrence of 30 d MACE in patients with acute chest pain was 0.901, which was significantly higher than 0.720 and 0.758 of single detection. This revealed that the HEART score combined with hs-CRP could better predict the occurrence of 30 d MACE in patients with acute chest pain and can improve sensitivity and specificity.

## 5. Conclusion

In conclusion, the HEART score combined with hs-CRP can better predict the occurrence of 30 d MACE in patients with acute chest pain, which is helpful for assisting clinical treatment decision-making.

## Figures and Tables

**Figure 1:** Predictive value of different indicators for 30 d MACE in patients with acute chest pain (the ROC curve above the reference line represented its diagnostic value, and the closer the curve to the upper left corner of the graph, the greater the diagnostic value).

**Table 1:** HEART scoring system.

Projects	Score
History	
Highly suspicion	2
Moderate suspicion	1
Mild suspicion or exclusion	0
ECG	
Significant depression or elevation of the ST segment	2
Nonspecific repolarization abnormalities	1
Bundle branch conduction block	1
Left ventricular hypertrophy	1
Normal	0
Age (years)	
>65	2
45∼65	1
<45	0
Risk factors (including diabetes, smoking, hypertension, hyperlipidemia, obesity, family history of coronary artery disease)	
>3 coronary heart disease risk factors or history of atherosclerosis treatment	2
1 or 2	1
0	0
Troponin (normal value ≤ 0.1 *μ*g/L)	
>2 times the upper limit of the normal value	2
1∼2 times the upper limit of the normal value	1
≤Upper limit of the normal value	0

**Table 2:** Occurrence of 30 d MACE in patients with different HEART scores.

Group	Number of cases	Incidence of MACE
HEART low-risk group	20	0 (0.00%)
HEART moderate-risk group	44	1 (2.27%)
HEART high-risk group	39	7 (17.95%)
*χ* ^2^ value		9.182
*P* value		0.010

**Table 3:** Comparison of clinical data between the two groups.

Projects	Non-MACE group (*n* = 95)	MACE group (*n* = 8)	*t*/*χ*^2^ value	*P* value
Age (years)	65.36 ± 4.71	68.88 ± 3.59	2.060	0.042
Male	52 (54.74%)	5 (62.50%)	0.180	0.671
Body mass index (kg/m^2^)	23.96 ± 3.14	23.56 ± 2.86	0.672	0.503
History of smoking	35 (36.84%)	4 (50.00%)	0.543	0.461
History of alcoholism	28 (29.47%)	3 (37.50%)	0.226	0.635
History of hypertension	61 (64.21%)	6 (75.00%)	0.378	0.539
History of diabetes	22 (23.16%)	3 (37.50%)	0.826	0.364
History of hyperlipidemia	24 (25.26%)	2 (25.00%)	0.001	0.987
History of coronary heart disease	46 (48.42%)	4 (50.00%)	0.007	0.932
Admission systolic blood pressure (mmHg)	140.31 ± 20.12	137.88 ± 20.27	0.327	0.743
Admission diastolic blood pressure (mmHg)	79.59 ± 15.69	78.87 ± 13.40	0.125	0.900
Admission heart rate (beats/min)	81.31 ± 11.90	81.13 ± 11.49	0.041	0.967
HEART score (points)	3.57 ± 0.75	7.50 ± 0.87	14.066	<0.001
hs-CRP (mg/L)	3.87 ± 0.40	5.98 ± 0.39	14.353	<0.001

**Table 4:** Risk factors for 30 d MACE in patients with acute chest pain.

Projects	B Value	SE value	Wald's value	OR value	95% CI	*P* value
Age	0.166	0.084	3.892	0.847	0.718∼1.009	0.050
HEART score	1.521	0.628	5.865	4.576	1.336∼15.666	0.015
hs-CRP	3.112	1.119	7.735	22.464	2.507∼21.329	0.005

**Table 5:** Predictive value of different indicators for 30 d MACE in patients with acute chest pain.

Variable	AUC	Standard error	*P* value	Asymptotic 95% CI		Youden index	Best cutoff value	Sensitivity (%)	Specificity (%)
				Lower limit	Upper limit				
HEART score	0.720	0.086	0.039	0.553	0.888	0.443	4.93 (points)	87.5	56.8
hs-CRP	0.758	0.086	0.016	0.589	0.927	0.383	4.65 (mg/L)	62.5	75.8
HEART score + hs-CRP	0.901	0.052	0.001	0.799	1.000	0.676	—	75.0	92.6

## Data Availability

All data included in this study are available upon request from the corresponding author.
